# The *PARK2* Mutation Associated with Parkinson's Disease Enhances the Vulnerability of Peripheral Blood Lymphocytes to Paraquat

**DOI:** 10.1155/2020/4658109

**Published:** 2020-09-21

**Authors:** Fengyu Ming, Jieqiong Tan, Lixia Qin, Hainan Zhang, Jianguang Tang, Xuling Tan, Chunyu Wang

**Affiliations:** ^1^Department of Neurology, The Second Xiangya Hospital, Central South University, Changsha, Hunan 410011, China; ^2^Department of Neurology, The First People's Hospital of Huaihua City, Hunan 418000, China; ^3^Center for Medical Genetics, School of Life Sciences, Central South University, Changsha, Hunan 410078, China; ^4^Department of Medical Genetics, The Second Xiangya Hospital, Central South University, Changsha, Hunan 410011, China

## Abstract

Parkinson's disease (PD) is the second most common neurodegenerative disease in middle-aged and elderly people. However, the etiology and pathogenesis of PD are still unclear and there is a lack of reliable biomarkers for early molecular diagnosis. Parkin (encoded by *PARK2*) is a ubiquitin E3 ligase that participates in mitochondrial homeostasis, the ubiquitin-proteasome pathway, oxidative stress response, and cell death pathways, which are involved in the pathogenesis of PD. However, Parkin is also expressed in peripheral blood lymphocytes (PBLs). In this study, permanent lymphocyte lines were established from the peripheral blood of sporadic PD (sPD) patients, *PARK2* mutation carriers, and healthy controls. Reactive oxygen species (ROS), function of the mitochondrial respiratory chain complex I, and apoptosis were analyzed in the PBLs. There was no significant difference in ROS, mitochondrial respiratory chain complex I, and apoptosis between the experimental groups and the control group without paraquat treatment. Compared with the control group of healthy subjects, we found an increase of ROS (control 100 ± 0, sPD 275.53 ± 79.11, and C441R 340 ± 99.67) and apoptosis, as well as a decline in the function of mitochondrial respiratory chain complex I in PBLs of *PARK2* mutation carriers and sPD after the treatment of paraquat (control 0.65 ± 0.08, sPD 0.44 ± 0.08, and C441R 0.32 ± 0.08). Moreover, overexpression of the wild-type (WT) *PARK2* in HeLa cells and immortalized PBLs could rescue mitochondrial function and partially inhibit apoptosis following paraquat treatment, while the C441R mutation could not. Thus, ROS levels, activity of mitochondrial respiratory chain complex I, and apoptosis of PBLs are potential diagnostic biomarkers of PD.

## 1. Introduction

Parkinson's disease (PD) is the second most common neurodegenerative disease after Alzheimer's disease (AD), with more than six million estimated cases in 2016 worldwide [1–3]. The overall prevalence of PD in industrialized countries is generally estimated at 0.3%, but it increases with age, from 1-2% at ages of 55-65 to more than 4% at ages of 85-89 [4]. Clinical symptoms of PD include bradykinesia, muscle rigidity, resting tremor, and postural instability, as well as increased susceptibility to memory impairment and behavioral alterations, including sleep abnormalities, depression, constipation, fatigue, and anxiety [3]. Pathologically, PD is characterized by the progressive loss of dopaminergic neurons in the *substantia nigra pars* compacta and the formation of abnormal protein aggregates in the surviving neurons, called Lewy bodies (LB) [5]. Although the etiology of PD is not clear, it is thought to be related to the environment, aging, and genetic predisposition [6–9].

Paraquat (1,1′-dimethyl-4,4′-bipyridine) is an important member of the bipyridylium family of broad-spectrum herbicides that are used in several crops including apples, cotton, beans, and sugarcane [10]. Paraquat crosses the blood-brain barrier via neutral amino acid transporters, preferentially targets the nigrostriatal pathway, inhibits the mitochondrial complex I, undergoes redox cycling, and produces superoxide radicals [11, 12]. An epidemiological study showed that exposure to paraquat strongly increases the risk of PD in humans [13]. In the experiment, paraquat has also been linked to the production of reactive oxygen species (ROS), oxidative stress, and aggregation of *α*-synucleins in dopaminergic neurons, although the mechanism by which paraquat affects dopaminergic neurons is not fully understood [12].

The *PARK2* (also known as *PRKN*/*PARKIN*) mutation causes the second most common form of familial PD and accounts for the majority of autosomal recessive PD (ARPD) cases, including both autosomal recessive juvenile PD (ARJPD) and late-onset PD (LOPD) [14–17]. Research showed that nearly 50% of ARJPD cases older than 25 and up to 7% of ARJPD cases ages 30-35 years carry mutations in *PARK2* [18, 19]. Several mutations in *PARK2* have been identified, including R42P, A46P, K211N, C212Y, C253Y, C289G, and C441R [20–24]. The *PARK2* encodes Parkin, which may directly cause mitochondrial dysfunction and was suggested to function as a multipurpose neuroprotective agent against a variety of toxic insults, including mitochondrial poisons, and is considered to be critical for the survival of dopaminergic neurons in mice [25]. Previous findings suggested that the absence of Parkin and PINK1 could increase the vulnerability of dopaminergic neurons to the effects of exogenous environmental stressors [26]. Mutations of *PARK2* impair its targeting to depolarized mitochondria and further inhibit mitophagy [20].

In spite of these earlier findings, there are no studies investigating whether *PARK2* mutations, and especially C441R, can increase the vulnerability of humans PBLs to environmental toxins. Here, we collected PBLs from 5 PD patients with *PARK2* C441R mutation, 5 cases of sporadic PD (sPD) without any known mutations and age-matched controls, to determine the vulnerability of PBLs carrying the *PARK2* C441R mutation to environmental toxins [27, 28].

## 2. Materials and Methods

### 2.1. Subjects

PD patients were clinically diagnosed in the Department of Neurology, Second Xiangya Hospital of Central South University, and Xiangya Hospital of Central South University, Hunan, China, according to the UK PD Society Brain Bank Clinical Diagnostic Criteria [29]. Genomic DNA was extracted from peripheral blood leukocytes using the QIAamp DNA Blood Mini Kit (Qiagen, Venlo, Germany). Mutation analysis of *PARK2*, PTEN-induced putative kinase 1 (*PINK1*), *DJ-1*, *ATP13A2*, *PLA2G6*, *CHCHD2*, *RAB39B*, *TMEM230*, and other genes associated with familial PD or early-onset PD (EOPD) was performed by multigene panel testing or Sanger sequencing. A total of 5 PD patients with *PARK2* C441R mutation and 5 sPD without the *PARK2* C441R mutation or other common pathogenic mutations were included in this study.

The disease onset age of the patients in the two groups was between 20 and 40 years old. The Hoehn-Yahr stage of PD patients in this study was 1–2.5 (Tables 1–3). The control group comprised healthy volunteers of the same age without PD or other neurological diseases. This study was approved by the Ethics Committee of the Second Xiangya Hospital, and written informed consent was obtained from all participants.

### 2.2. Isolation of Lymphocytes and Cell Culture

PBLs were isolated using a Ficoll-1077 (C-44010, Sigma) density gradient. Isolated PBLs were washed three times with PBS, suspended in RPMI 1640 (containing 10% FBS, 2 mM L-glutamine, and 1% penicillin/streptomycin), and cultivated at 37°C in a humidified atmosphere comprising 5% CO_2_. The HeLa cells were cultured in DMEM containing 10% FBS and 1% penicillin/streptomycin at 37°C in a humidified atmosphere comprising 5% CO_2_.

### 2.3. Cell Immortalization

The Lenti-SV40T lentivirus vector was diluted with fresh complete medium (1 : 1), and transfection was performed using the Lipofectamine™ 3000 Transfection Reagent (#L3000015, Invitrogen), according to the manufacturer's protocol. On the next day, the viral supernatant was removed and the appropriate complete growth medium was added to the cells. After 72 h of incubation at 37°C, the cells were subcultured and puromycin was added to select stable cell-lines. Following 10-15 days after selection, individual clones were picked and expanded.

### 2.4. Measurement of ROS

The generation of ROS was measured using the peroxide-sensitive fluorescent probe 2′7′ dichlorofluorescein diacetate (DCFH-DA) (#D6883, Sigma, USA). PBLs were treated with 1 mM paraquat for 24 h, collected, and washed them 2 times with PBS. Cells that underwent different treatments were incubated with DCFH-DA (10 *μ*M) for 30 min at 37°C in the dark. DCFH-DA was converted by intracellular esterases into DCFH, which was oxidized into the highly fluorescent dichlorofluorescein in the presence of ROS. The cells were mounted and visualized by confocal microscopy, and the fluorescence was measured using Fluoroskan Ascent at 488/525 nm. The intensity of DCFH-DA fluorescence was quantified densitometrically using Image J software (NIH; USA).

### 2.5. Mitochondrial Complex I Activity Assay

Mitochondrial complex I activity was measured using the Complex I Enzyme Activity Kit (#ab109721, Abcam, UK) following the manufacturer's directions. PBLs were treated with 1 mM paraquat for 24 h, harvested by centrifugation at 1000 g, and washed twice with ice-cold PBS. Mitochondria were isolated using the Mitochondria Isolation Kit (Abcam). Purified mitochondria were suspended in 500 *μ*L Buffer C and lysed for 30 min by adding the detergent provided in the kit. After centrifugation, the mitochondrial proteins were quantified using the Bradford assay, and mitochondrial lysates were adjusted to the same protein concentration (approximately 1 mg/ml). Serial dilutions were prepared in the incubation solution (Abcam CI Assay Kit). Complex I activity was measured using 200 *μ*L aliquots of the serial dilutions, each in triplicate, using the Molecular Devices VERSAmax microplate reader at 450 nm, with kinetic readings taken every 30 sec for 30 minutes. Activity was represented as mOD/min and normalized to the control group (defined as 1.00).

### 2.6. Measurement of Apoptosis

Apoptosis was measured using the Annexin V-FITC Apoptosis Detection Kit (#APOAF, Sigma). Briefly, collected cells were washed 2 times with PBS, after which 500 *μ*L of binding buffer, 5 *μ*L of Annexin V-FITC, and 10 *μ*L of propidium iodide were and incubated at 37°C for 5-15 min in the dark. The apoptosis rate of PBLs was quantified using a FACSCanto™ II (BD Biosciences, Franklin Lakes, NJ, USA).

### 2.7. Cytochrome C Release

Cells were lysed in buffer containing 250 mM sucrose, 20 mM HEPES, pH 7.5, 10 mM KCl, 1.5 mM MgCl2, 1 mM EGTA, 1 mM DTT, and protease inhibitor set (Roche diagnostic, Basel, Switzerland). The homogenates were centrifuged twice at 750 g for 10 min at 4°C, the resulting supernatants were centrifuged at 10 000 g for 15 min at 4°C, and the second supernatants were further centrifuged at 100 000 g for 1 h at 4°C. The remaining supernatants contained cytosolic proteins that were separated by SDS–PAGE on a 15% acrylamide gel for immunoblotting assays.

### 2.8. Immunoblotting Assays

Cells were washed with PBS and then lysed with ice-cold lysis buffer (50 mM Tris-HCl pH 7.5, 150 mM NaCl, 1 mM EDTA, 1% Triton X-100) supplemented with protease inhibitor cocktail (B14001; Biotool, Switzerland). After incubation on ice for 30 min, homogenates were centrifuged at 16,000 g for 15 min at 4°C. Supernatants were collected, and protein concentrations were determined using the BCA protein assay kit (#23227; Thermo Fisher Scientific, USA). Proteins were separated by SDS-PAGE and transferred to a PVDF membrane. After blocking nonspecific binding sites for 1 h with 10% nonfat milk, the blots were detected using primary antibodies against cytochrome C (#4280), cleaved caspase 9 (#52873), and actin (#3700) (All from Cell Signaling Technology, USA). Chemiluminescent bands were detected using a CCD camera (Amersham Imager 600; GE Healthcare, USA) and quantified densitometrically using Image J software (NIH, USA).

### 2.9. Immunohistochemical Staining

Cells grown on coverslips were fixed with 4% paraformaldehyde for 15 min, permeabilized with 0.1% Triton X-100 in PBS for 15 min, and blocked with 5% FBS in PBS for 2 h at room temperature. The fixed cells were then incubated with the primary antibody (TOM20 (#42406) and Myc-Tag (#2276); Cell Signaling Technology, USA) at 4°C overnight, followed by incubation with the secondary antibodies for 1 h at room temperature. Finally, the secondary antibodies were visualized by confocal microscopy.

### 2.10. Statistical Analysis

All the results were presented as means ± SD. Statistical analysis of the data was performed using Mann–Whitney *U* nonparametric tests. Differences with *p* < 0.05 were considered statistically significant.

## 3. Results

### 3.1. Lymphocytes from PD Patients Are More Vulnerable to Mitochondrial Damage and Apoptosis Induced by Paraquat

It has reported that Parkin is expressed in PBLs and Parkin mutations cause mitochondrial dysfunction [30]. Here, we detected the ROS levels of PBLs from health controls, sPD patients, and PD patients carried the *PARK2* C441R mutation after paraquat treatment. We found that the ROS levels were significantly increased in PBLs from both sPD patients and those with the *PARK2* C441R mutation compared to healthy controls (control 100 ± 0, sPD 275.53 ± 79.11, and C441R 340 ± 99.67; Figures 1(a) and 1(b)). Moreover, compared with the controls, the activity of mitochondrial complex I was decreased in PBLs from the sPD patients, and even more in patients with the Parkin mutation (control 0.65 ± 0.08, sPD 0.44 ± 0.08, and C441R 0.32 ± 0.08; Figure 1(c)). In addition, we examined the apoptosis levels via Annexin V-FITC staining and flow cytometry. The results showed an increase of apoptosis in PBLs from sPD and Parkin mutation patients compared with healthy controls (Figure 1(d)).

### 3.2. Overexpression of WT Parkin but Not the C441 Mutant Protected HeLa Cells and Immortalized PBLs from Paraquat-Induced Mitochondrial Damage and Apoptosis

Carbonyl cyanide m-chlorophenylhydrazone (CCCP) was used as a positive control. Parkin WT or C441R was expressed in HeLa cells. CCCP treatment caused a decrease in membrane potential and recruited Parkin to the mitochondrial outer membrane. The colocalization analysis showed that WT Parkin, but not the C441R mutant was recruited to damaged mitochondria after paraquat treatment (Parkin WT+DMSO 6.08 ± 3.79%, Parkin WT+CCCP 62.49 ± 16.47%, Parkin WT+paraquat 45.33 ± 14.84%, Parkin C441Rmutant+paraquat 7.09 ± 3.85%; Figures 2(a) and 2(b)).

To further understand the effects of Parkin on apoptosis, we transfected both HeLa cells and immortalized PBLs with either empty vector, Parkin WT, or C441R mutant Parkin, followed by paraquat treatment.

In HeLa cells, the control treatment induced 3.48 ± 1.61%apoptosis, empty vector+paraquat 45.68 ± 6.95%, WT+paraquat 24.98 ± 5.70%, C441R+paraquat 49.3 ± 10.90% (Figure 2(c)). In immortalized PBLs: the control treatment induced 2.05 ± 0.77% apoptosis, empty vector+paraquat 54.78 ± 10.94%, WT+paraquat 29.44 ± 8.12%, and C441R+paraquat 55.24 ± 7.72% (Figure 2(d)). These results indicated that overexpression of WT Parkin but not the C441R mutation rescued HeLa cells and immortalized PBLs from apoptosis induced by paraquat treatment. Moreover, the levels of cytochrome C and cleaved caspase 9 were determined by western blot analysis. Compared to the empty vector, overexpression of WT Parkin resulted in a significant decrease of cytochrome C and cleaved caspase 9 levels after paraquat treatment, but the Parkin C441R mutant did not (Figure 2(e)).

## 4. Discussion

The question of the contributions of genetic and environmental factors in the etiology of PD has been puzzling researchers for a long time. There is still no definite answer as to how the factors such as environment, heredity, and aging are combined and which are dominant or secondary. Genetic factors may increase the risk of sPD, while environmental factors may aggravate hereditary PD [31, 32].

The results of this study indicate that after paraquat treatment, the mitochondrial complex I activity of PBLs from sPD patients, as well as patients with the C441R mutation group and the healthy controls decreased, while the ROS levels and lymphocyte apoptosis increased significantly. This suggests that environmental factors (paraquat) may induce apoptosis of PBLs in healthy people and PD patients by causing mitochondrial dysfunction, which was in agreement with previous studies [33]. In addition, ROS levels and mitochondrial complex I activity decreased and apoptosis increased significantly in the sPD and mutated Parkin groups compared with the control group, especially in the latter. Previous studies suggested that paraquat could reduce the survival of dopaminergic neurons in the substantia nigra striatum of PD model mice, indicating that PD increased the sensitivity of cells to neurotoxins, leading to more obvious mitochondrial dysfunction and aggravating apoptosis [34]. This mechanism can explain why the cells derived from PD patients were more sensitive to paraquat than those from healthy controls. In addition, as a ubiquitin ligase (E3), Parkin protein is involved in mitochondrial autophagy, maintenance of mitochondrial function, and degradation of misfolded proteins, which plays an important role in maintaining the integrity of organelles [35]. Accordingly, an abnormal structure or function of Parkin protein may lead to mitochondrial dysfunction [36, 37]. Parkin protein consists of three domains, named UBL, RBR, and RING0. The E3 ubiquitin ligase activity mainly depends on the RBR domain, which recruits the E2 ubiquitin-binding enzyme. The C441R mutation is located in the RING2 domain, and previous studies suggested that it can change its structure, which may affect its interaction with the E2 ubiquitin-binding enzyme and lead to mitochondrial dysfunction [38]. The results of the immortalized leucocytes from the sPD group and Parkin C441R mutation group indicate that the mutation made the cells more sensitive to the effects of environmental toxins, leading to increased mitochondrial dysfunction and apoptosis.

The localization of Parkin to the mitochondria was evident in HeLa cells transfected with Parkin WT after paraquat and CCCP treatment compared with the control group. The reason may be that environmental toxins such as paraquat activate the Parkin-PINK1 pathway, which causes mitochondrial autophagy [39]. PINK1 is a ubiquitous protein kinase, and its N-terminal contains a mitochondrial localization signal, which targets it to the mitochondria. Under normal conditions, PINK1 is located in mitochondria, cut by hydrolytic enzymes, and releasesd into the cytoplasm for rapid degradation. When the mitochondrial membrane potential (MMP) is reduced, for example by exposure to the mitochondrial decoupling agent CCCP, PINK1 cannot be processed normally and cannot enter mitochondria through the translocation complex between the mitochondrial inner and outer membranes. This leads to the aggregation of PINK1 protein on the outer membrane of the mitochondria, activates and recruits Parkin protein, and finally causes mitochondrial autophagy [40]. However, after paraquat treatment, the localization of Parkin to mitochondria was significantly different in the HeLa cells expressing WT and mutant Parkin. The reason may be that C441R leads to a folding defect in the protein structure, causing abnormal localization of Parkin [41–43].

Additionally, our results showed that the apoptosis rate of HeLa cells and immortalized PBLs transfected with WT Parkin was significantly lower than that of the vector controls and C441R mutant groups. Similarly, the levels of cytochrome C and cleaved caspase-9 in HeLa cells transfected with WT Parkin were significantly lower than in the vector control and C441R mutant groups. This may be due to the protective effect of Parkin protein, which can reverse or reduce apoptosis caused by paraquat [25, 44]. The experiments indicate that stratification of different groups of patients by assessing peripheral blood samples may provide a novel and facile diagnostic biomarker.

Nevertheless, the experiments have limitations that must be considered when interpreting the results. The number of subjects included in this study was small, and a larger sample size is needed to confirm the results. Furthermore, it may be useful to measure time-series after treatment with paraquat for 24 h. Moreover, other experiments for measuring complex I activity and apoptosis may be needed to reconfirm our results. In addition, the role of Parkin mutation in the pathogenesis of PD involves multiple mechanisms. This research was limited to discussing the effect of Parkin mutation on mitochondrial function in combination with environmental toxins, and there was no in-depth study on the mechanism, which still has some limitations. In addition, although peripheral blood lymphocytes have limited similarities with dopaminergic neurons in some aspects, more studies are needed to confirm whether they can reflect the state of central dopaminergic neurons. In conclusion, the measurement of mitochondrial function and apoptosis of PBLs may indeed provide certain clues for the early diagnosis of PD.

## Figures and Tables

**Figure 1:** Lymphocytes in PD patients are more sensitive to mitochondrial damage and apoptosis induced by paraquat. (a) After treatment with 1 mM paraquat, the ROS levels of immortalized lymphocytes were detected by stained with DCFH-DA (green). The nuclei were counter-stained with Hoechst 33342 (blue). (b) Quantification of DCFH-DA. (c) Quantification of the activity of mitochondrial complex I of immortalized lymphocytes from controls, sporadic PD patients, and PD patients with Parkin mutantion, following treatment with DMSO (control) or paraquat. (d) Quantification of apoptosis of immortalized lymphocytes from controls, sporadic PD patients, and PD patients with Parkin mutation, following treatment with DMSO or paraquat. *n* = 3, ∗*p* < 0.05; ∗∗*p* < 0.01; ∗∗∗*p* < 0.001.

**Figure 2:** Overexpression of WT Parkin, but not the C441 mutant, protected HeLa cells and immortalized PBLs against paraquat-induced mitochondrial damage and apoptosis. (a) HeLa cells cotransfected with mitochondrial marker TOM20 (red) and WT Parkin or the C441R mutant (green) were treated with 1 mM paraquat (left panel). (b) Quantification of cells displaying Parkin co-localization with mitochondria (right panel). (c, d) Quantification of apoptosis in HeLa cells and immortalized lymphocytes transfected with empty vector, Parkin WT, or C441R mutant after paraquat treatment. (e) Cytosolic cytochrome *C* and cleaved caspase 9 levels in immortalized lymphocytes transfected with empty vector, Parkin WT, or C441R mutant after paraquat treatment, detected by western blot analysis. *n* = 3, ∗*p* < 0.05; ∗∗*p* < 0.01.

**Table 1:** Clinical features of sporadic patients.

Clinical feature	Patient 1	Patient 2	Patient 3	Patient 4	Patient 5
Sex	Woman	Woman	Man	Man	Man
Age at disease onset (years)	34	31	33	30	36
Disease duration (years)	3	2	5	6	5
Bradykinesia	+	+	+	+	+
Rigidity	+	+	+	+	+
Resting tremor	—	—	+	+	—
Postural tremor	—	—	—	+	—
Shuffling gait	—	—	+	—	+
Postural instability	—	—	—	—	—
Hyperreflexia	—	—	—	—	—
Diurnal fluctuations	—	—	—	+	—
Foot dystonia	—	—	—	—	—
Hoehn and Yahr stage at last examination (off state)	1	1	2	2	2
UPDRS III score at last exam (off state)	13	17	22	24	20

**Table 2:** Clinical features of patients with *PARK2* C441R mutation.

Clinical feature	Patient 1	Patient 2	Patient 3	Patient 4	Patient 5
Sex	Woman	Man	Man	Man	Man
Age at disease onset (years)	23	34	32	20	40
Disease duration (years)	2	2	6	7	10
Bradykinesia	+	+	+	+	+
Rigidity	+	+	+	+	+
Resting tremor	—	—	+	+	+
Postural tremor	—	—	+	+	—
Shuffling gait	—	—	—	+	+
Postural instability	—	—	—	+	—
Hyperreflexia	—	+	—	+	—
Diurnal fluctuations	—	—	—	+	+
Foot dystonia	—	+	—	+	+
Hoehn and Yahr stage at last examination (off state)	1	1	2	2.5	2.5
UPDRS III score at last exam (off state)	12	15	19	22	27

**Table 3:** Clinical features of patients in the study sample.

Clinical feature	Patients without mutation	Patients with Parkin mutation
Number	5 [3/2]^a^	5 [4/1]^a^
Age at disease onset (years)	32.80 ± 2.39	29.80 ± 8.20
Disease duration (years)	4.20 ± 1.64	5.4 ± 3.44
Bradykinesia	5 (100)^b^	5 (100)^b^
Rigidity	5 (100)^b^	5 (100)^b^
Resting tremor	2 (40)^b^	3 (66.7)^b^
Postural tremor	1 (20)^b^	2 (40)^b^
Shuffling gait	2 (40)^b^	2 (40)^b^
Postural instability	0 (0)^b^	1 (20)^b^
Hyperreflexia	0 (0)^b^	2 (40)^b^
Diurnal fluctuations	1 (20)^b^	2 (40)^b^
Foot dystonia	0 (0)^b^	3 (66.7)^b^
UPDRS III score at last exam (off state)	19.20 ± 4.32	19.00 ± 5.87

^a^Values in square brackets indicate *M*/*W* ratios. ^b^Values in parentheses indicate percentages.

## Data Availability

The data used to support the findings of this study are available from the corresponding author upon request.

## References

[1] Dorsey E. R., Elbaz A., Nichols E. (2018). Global, regional, and national burden of Parkinson's disease, 1990–2016: a systematic analysis for the global burden of disease study 2016. *Lancet Neurology*.

[2] Shtilbans A., Henchcliffe C. (2012). Biomarkers in Parkinson's disease: an update. *Current Opinion in Neurology*.

[3] Savitt J. M., Dawson V. L., Dawson T. M. (2006). Diagnosis and treatment of Parkinson disease: molecules to medicine. *Journal of Clinical Investigation*.

[4] Ibanez L., Dube U., Saef B. (2017). Parkinson disease polygenic risk score is associated with Parkinson disease status and age at onset but not with alpha-synuclein cerebrospinal fluid levels. *BMC Neurology*.

[5] Charvin D., Medori R., Hauser R. A., Rascol O. (2018). Therapeutic strategies for Parkinson disease: beyond dopaminergic drugs. *Nature Reviews Drug Discovery*.

[6] Dauer W., Przedborski S. (2003). Parkinson's disease: mechanisms and models. *Neuron*.

[7] de Lau L. M., Breteler M. M. (2006). Epidemiology of Parkinson's disease. *Lancet Neurology*.

[8] Bellou V., Belbasis L., Tzoulaki I., Evangelou E., Ioannidis J. P. A. (2016). Environmental risk factors and Parkinson's disease: an umbrella review of meta-analyses. *Parkinsonism & Related Disorders*.

[9] Vlaar T., Kab S., Schwaab Y., Frery N., Elbaz A., Moisan F. (2018). Association of Parkinson’s disease with industry sectors: a French nationwide incidence study. *European Journal of Epidemiology*.

[10] Vaccari C., el Dib R., de Camargo J. L. V. (2017). Paraquat and Parkinson's disease: a systematic review protocol according to the OHAT approach for hazard identification. *Systematic Reviews*.

[11] Kumar A., Leinisch F., Kadiiska M. B., Corbett J., Mason R. P. (2016). Formation and implications of alpha-synuclein radical in maneb- and paraquat-induced models of Parkinson's disease. *Molecular Neurobiology*.

[12] Reczek C. R., Birsoy K., Kong H. (2017). A CRISPR screen identifies a pathway required for paraquat-induced cell death. *Nature Chemical Biology*.

[13] Franco R., Li S., Rodriguez-Rocha H., Burns M., Panayiotidis M. I. (2010). Molecular mechanisms of pesticide-induced neurotoxicity: relevance to Parkinson's disease. *Chemico-Biological Interactions*.

[14] Corti O., Lesage S., Brice A. (2011). What genetics tells us about the causes and mechanisms of Parkinson's disease. *Physiological Reviews*.

[15] Zhao Y., Qin L., Pan H. (2020). The role of genetics in Parkinson's disease: a large cohort study in Chinese mainland population. *Brain*.

[16] Koyano F., Okatsu K., Kosako H. (2014). Ubiquitin is phosphorylated by PINK1 to activate parkin. *Nature*.

[17] Hou X., Fiesel F. C., Truban D. (2018). Age- and disease-dependent increase of the mitophagy marker phospho-ubiquitin in normal aging and Lewy body disease. *Autophagy*.

[18] Hattori N., Mizuno Y. (2017). Twenty years since the discovery of the parkin gene. *Journal of Neural Transmission (Vienna)*.

[19] Klein C., Lohmann-Hedrich K., Rogaeva E., Schlossmacher M. G., Lang A. E. (2007). Deciphering the role of heterozygous mutations in genes associated with parkinsonism. *Lancet Neurology*.

[20] Narendra D. P., Jin S. M., Tanaka A. (2010). PINK1 is selectively stabilized on impaired mitochondria to activate Parkin. *PLoS Biology*.

[21] Gonzalez-Casacuberta I., Juarez-Flores D. L., Moren C., Garrabou G. (2019). Bioenergetics and autophagic imbalance in patients-derived cell models of Parkinson disease supports systemic dysfunction in neurodegeneration. *Frontiers in Neuroscience*.

[22] Bekris L. M., Mata I. F., Zabetian C. P. (2010). The genetics of Parkinson disease. *Journal of Geriatric Psychiatry and Neurology*.

[23] Hedrich K., Eskelson C., Wilmot B. (2004). Distribution, type, and origin of Parkin mutations: review and case studies. *Movement Disorders*.

[24] Hedrich K., Marder K., Harris J. (2002). Evaluation of 50 probands with early-onset Parkinson's disease for Parkin mutations. *Neurology*.

[25] Pickrell A. M., Youle R. J. (2015). The roles of PINK1, parkin, and mitochondrial fidelity in Parkinson's disease. *Neuron*.

[26] Zeng X. S., Geng W. S., Jia J. J., Chen L., Zhang P. P. (2018). Cellular and molecular basis of neurodegeneration in Parkinson disease. *Frontiers in Aging Neuroscience*.

[27] Guo J. F., Xiao B., Liao B. (2008). Mutation analysis of Parkin, PINK1, DJ-1 and ATP13A2 genes in Chinese patients with autosomal recessive early-onset Parkinsonism. *Movement Disorders*.

[28] Guo J. F., Dong X. L., Xu Q. (2015). Exon dosage analysis of parkin gene in Chinese sporadic Parkinson's disease. *Neuroscience Letters*.

[29] Litvan I., Bhatia K. P., Burn D. J. (2003). Movement disorders society scientific issues committee report: SIC task force appraisal of clinical diagnostic criteria for Parkinsonian disorders. *Movement Disorders*.

[30] Kasap M., Akpinar G., Sazci A., Idrisoglu H. A., Vahaboglu H. (2009). Evidence for the presence of full-length PARK2 mRNA and Parkin protein in human blood. *Neuroscience Letters*.

[31] Schapira A. H. V., Gu M., Taanman J. W. (1998). Mitochondria in the etiology and pathogenesis of Parkinson's disease. *Annals of Neurology*.

[32] Sherer T. B., Betarbet R., Greenamyre J. T. (2002). Environment, mitochondria, and Parkinson's disease. *The Neuroscientist*.

[33] Rio M. J., Velez-Pardo C. (2008). Paraquat induces apoptosis in human lymphocytes: protective and rescue effects of glucose, cannabinoids and insulin-like growth factor-1. *Growth Factors*.

[34] Thiruchelvam M., McCormack A., Richfield E. K. (2003). Age-related irreversible progressive nigrostriatal dopaminergic neurotoxicity in the paraquat and maneb model of the Parkinson's disease phenotype. *European Journal of Neuroscience*.

[35] Arkinson C., Walden H. (2018). Parkin function in Parkinson's disease. *Science*.

[36] Cornelissen T., Vilain S., Vints K., Gounko N., Verstreken P., Vandenberghe W. (2018). Deficiency of parkin and PINK1 impairs age-dependent mitophagy in Drosophila. *eLife*.

[37] Cornelissen T., Verstreken P., Vandenberghe W. (2018). Imaging mitophagy in the fruit fly. *Autophagy*.

[38] Wenzel D. M., Klevit R. E. (2012). Following Ariadne's thread: a new perspective on RBR ubiquitin ligases. *BMC Biology*.

[39] Hamacher-Brady A., Brady N. R. (2016). Mitophagy programs: mechanisms and physiological implications of mitochondrial targeting by autophagy. *Cellular and Molecular Life Sciences*.

[40] McWilliams T. G., Muqit M. M. (2017). PINK1 and Parkin: emerging themes in mitochondrial homeostasis. *Current Opinion in Cell Biology*.

[41] Fedorowicz M. A., Vries-Schneider R. L. A., Rüb C. (2013). Cytosolic cleaved PINK1 represses Parkin translocation to mitochondria and mitophagy. *Embo Reports*.

[42] Lazarou M., Narendra D. P., Jin S. M., Tekle E., Banerjee S., Youle R. J. (2013). PINK1 drives Parkin self-association and HECT-like E3 activity upstream of mitochondrial binding. *The Journal of Cell Biology*.

[43] Hampe C., Ardila-Osorio H., Fournier M., Brice A., Corti O. (2006). Biochemical analysis of Parkinson’s disease-causing variants of Parkin, an E3 ubiquitin–protein ligase with monoubiquitylation capacity. *Human Molecular Genetics*.

[44] Spratt D. E., Walden H., Shaw G. S. (2014). RBR E3 ubiquitin ligases: new structures, new insights, new questions. *Biochemical Journal*.

